# Drug-Drug Interactions Prediction Using Fingerprint Only

**DOI:** 10.1155/2022/7818480

**Published:** 2022-05-09

**Authors:** Bing Ran, Lei Chen, Meijing Li, Yujuan Han, Qi Dai

**Affiliations:** ^1^College of Information Engineering, Shanghai Maritime University, Shanghai 201306, China; ^2^College of Life Sciences, Zhejiang Sci-Tech University, Hangzhou 310018, China

## Abstract

Combination drug therapy is an efficient way to treat complicated diseases. Drug-drug interaction (DDI) is an important research topic in this therapy as patient safety is a problem when two or more drugs are taken at the same time. Traditionally, in vitro experiments and clinical trials are common ways to determine DDIs. However, these methods cannot meet the requirements of large-scale tests. It is an alternative way to develop computational methods for predicting DDIs. Although several previous methods have been proposed, they always need several types of drug information, limiting their applications. In this study, we proposed a simple computational method to predict DDIs. In this method, drugs were represented by their fingerprint features, which are most widely used in investigating drug-related problems. These features were refined by three models, including addition, subtraction, and Hadamard models, to generate the representation of DDIs. The powerful classification algorithm, random forest, was picked up to build the classifier. The results of two types of tenfold cross-validation on the classifier indicated good performance for discovering novel DDIs among known drugs and acceptable performance for identifying DDIs between known drugs and unknown drugs or among unknown drugs. Although the classifier adopted a sample scheme to represent DDIs, it was still superior to other methods, which adopted features generated by some advanced computer algorithms. Furthermore, a user-friendly web-server, named DDIPF (http://106.14.164.77:5004/DDIPF/), was developed to implement the classifier.

## 1. Introduction

Drugs are deemed as an efficient way to treat different diseases. However, some diseases are so complex that it is almost impossible to treat them with a single drug because several targets are involved. In view of this, combination drug therapy is proposed, which can improve drug efficacy and reduce drug resistance [1]. This method should be carefully used because some drugs can interact with others when they are taken at the same time. These drug-drug interactions (DDIs) may cause a serious problem in patient safety [2, 3]. On the other hand, the safety problem caused by unexpected DDIs can lead to the withdrawal of drugs from the market, bringing great risks to pharmaceuticals companies. Thus, the correct determination of DDIs is important in the drug research area. Traditional in vitro experiments and clinical trials can solidly complete this task. However, these methods also have some shortcomings, such as low efficiency and high cost. It is necessary to design quick and reliable methods for predicting DDIs.

In recent years, with the development of high-throughput methods, more and more properties of drugs have been discovered, which are stored in some online databases, such as DrugBank [4, 5], KEGG [6], and STITCH [7]. By analyzing these abundant properties, investigators can discover novel features of drugs. However, how to analyze such huge properties is a problem. Fortunately, lots of newly proposed computer algorithms provide strong technical support. For predicting DDIs, several computational methods have been proposed. Although these methods cannot output assured results, they can provide new clues for discovering novel DDIs. Most computational methods always deeply analyze current known DDIs and form patterns to predict latent DDIs. To date, several types of computer algorithms have been adopted to design quick and reliable methods for predicting DDIs. Among them, machine learning algorithms play essential roles [8–13]. For example, Kastrin et al. [9] designed topological and semantic feature similarities, which were learnt by five classification algorithms to construct the classifier. Cheng and Zhao [10] set up a support vector machine (SVM) model to predict DDIs, which adopted features derived from the Simplified Molecular Input Line Entry System (SMILES) and side effect similarities of the two drugs. Chen et al. [11] proposed a nearest neighbor algorithm- (NNA-) based model to identify DDIs, which designed a scheme to measure the similarity of two drug pairs. Besides the machine learning-based methods, several other methods, such as deep learning-based [14–17], network-based [18–20], and text mining-based [21–23], were also proposed to identify DDIs. Most previous methods adopted several types of drug properties, indicating that they cannot provide the result if these properties of the input drug are not available. This fact limits the applications of these methods.

In this study, we proposed a simple computational method to predict DDIs. For wide applications of the method, drugs were only represented by their fingerprint features, which can be easily obtained if their SMILES formats are available. Based on drug fingerprint features, three models, including addition, subtraction, and Hadamard models, were designed to generate features of each drug pair. The powerful classification algorithm, random forest (RF) [24], was used to construct the method. After trying all combinations of features produced by three models, we found the classifier using features generated by addition and subtraction models was the best for predicting DDIs among known drugs, and another classifier using features generated by addition and Hadamard models was proper to identify DDIs between known drugs and unknown ones or among unknown drugs. Although the method adopted the generally used fingerprint features, it was superior to some methods, which used some advanced drug features.

## 2. Materials and Methods

### 2.1. Materials

The 6185 experimental validated drugs were retrieved from DrugBank (https://go.drugbank.com/) [4, 5], a public dataset containing information on drugs and drug targets. Because we used fingerprints of drugs to conduct this investigation, drugs that cannot extract their fingerprints were removed, resulting in 6175 drugs. Then, we downloaded the DDIs involving these 6175 drugs from DrugBank, obtaining 37496 DDIs. These DDIs covered 722 drugs. As the obtained DDIs have been solidly validated, they were termed positive samples in this study.

To construct a binary classifier, negative samples were also necessary. They were produced in the following manner. From the 772 drugs involved in positive samples, randomly pick up two different drugs. If they cannot comprise a positive sample, they were picked up as a negative sample. This procedure was conducted several times until the number of different negative samples was equal to that of positive samples. The obtained negative samples and above-mentioned positive samples were combined to constitute a dataset, denoted by *D*.

### 2.2. Drug Representation with Its Fingerprints

It is an essential problem to represent drugs with numbers when constructing efficient models for dealing with drug-related problems. The SMILES [25] format is the most widely accepted scheme to represent a drug. It is a line notation with ASCII strings to represent molecules and reactions. With this representation, the fingerprints can be extracted for a given fingerprint type. Here, we used RDKit (http://www.rdkit.org) to extract ECFP_4 fingerprints [26] for each investigated drug. Generally, the fingerprints of one drug are represented by a binary vector, where each component denotes one fingerprint. The component is set to one if the drug has the corresponding fingerprint of this component. In this way, each of 772 drugs *d* was encoded into a 1024-D vector, formulated by

(1) $$\begin{array}{c} F\left(d\right)={\left[f_{1},f_{2},\cdots ,f_{1024}\right]}^{T}. \end{array}$$

### 2.3. DDI Representation

For a DDI *D* = [*d*_1_, *d*_2_], where *d*_1_ and *d*_2_ were two drugs, features can be obtained from their fingerprint vectors *F*(*d*_1_) and *F*(*d*_2_). Since there was no sequence information in the pair of *d*_1_ and *d*_2_, that is, [*d*_1_, *d*_2_] = [*d*_2_, *d*_1_], it was not rigorous by directly combining *F*(*d*_1_) and *F*(*d*_2_) into one vector because it was a problem of which fingerprint vector should be put in the front of the final vector. In view of this, we adopted the following three schemes to fuse two fingerprint vectors into one vector, while the order information was not involved. To give a clear description, let us denote *F*(*d*_1_) and *F*(*d*_2_) by *F*(*d*_1_) = [*f*_1_^1^, *f*_2_^1^, ⋯,*f*_1024_^1^]^*T*^ and *F*(*d*_2_) = [*f*_1_^2^, *f*_2_^2^, ⋯,*f*_1024_^2^]^*T*^, respectively. The first one was the addition model, which fused *F*(*d*_1_) and *F*(*d*_2_) into a new vector *V*_*A*_(*D*) using the addition operation, formulated by

(2) $$\begin{array}{c} V_{A}\left(D\right)={\left[f_{1}^{1}+f_{1}^{2},f_{2}^{1}+f_{2}^{2},\cdots ,f_{1024}^{1}+f_{1024}^{2}\right]}^{T}. \end{array}$$

The second scheme was the subtraction model. *F*(*d*_1_) and *F*(*d*_2_) were fused into a new vector *V*_*S*_(*D*), defined by

(3) $$\begin{array}{c} V_{S}\left(D\right)={\left[\left|f_{1}^{1}-f_{1}^{2}\right|,\left|f_{2}^{1}-f_{2}^{2}\right|,\cdots ,\left|f_{1024}^{1}-f_{1024}^{2}\right|\right]}^{T}, \end{array}$$

where |·| represents the absolute operation. The last scheme was the Hadamard model, which fused *F*(*d*_1_) and *F*(*d*_2_) as follows:

(4) $$\begin{array}{c} V_{H}\left(D\right)={\left[f_{1}^{1}\cdot f_{1}^{2},f_{2}^{1}\cdot f_{2}^{2},\cdots ,f_{1024}^{1}\cdot f_{1024}^{2}\right]}^{T}. \end{array}$$

Through the above three schemes, each DDI can be represented by three vectors. In this study, we would try each combination to represent DDIs, thereby determining the optimum representation for predicting DDIs.

### 2.4. Random Forest

Besides efficient features, a proper classification algorithm is also important to construct a powerful classifier. In this study, we selected the classic classification algorithm, RF [24]. Such an algorithm is always a candidate for building models to tackle different biological or medical problems [27–32].

RF is a type of ensemble algorithm, which contains several decision trees. Two random selection procedures are involved to construct each decision tree. The first random selection is for samples. Given a dataset with *n* samples, randomly select *n* samples, with replacement, to constitute a new dataset, based on which a decision tree is built. The second random selection is for features. Selected features are used to split one node to extend the tree. Although the decision tree is a weak classification algorithm, RF is much more powerful [33].

This study used the RF program in scikit-learn (https://scikit-learn.org/) [34]. Default parameters were used to execute such a program. The number of decision trees was 100.

### 2.5. Cross-Validation Method

Cross-validation [35] is a widely used scheme to evaluate the performance of classifiers. This study also adopted such a method. Based on the composition of samples in this study, two types of cross-validation were designed to fully evaluate the performance of all constructed classifiers.

For the first type of cross-validation, DDIs were equally and randomly divided into *K* parts. Each part was singled out one by one to comprise the test dataset and the rest parts were combined to constitute the training dataset. The model based on the training dataset was applied to the test dataset. Accordingly, each DDI was tested exactly once.

The second type of cross-validation was quite different. It first divided drugs into *K* parts. Each part was singled out one by one to constitute the drug test dataset, whereas drugs in the rest nine parts were combined as the drug training dataset. From the original dataset, three datasets were constructed in this test, called the training dataset, One Drug In Train (ODIT) test dataset, and No Drug In Train (NDIT) test dataset. The training dataset included DDIs such that two drugs were all in the drug training dataset, the ODIT test dataset contained DDIs that one drug was in the drug training dataset and the other drug was in the drug test dataset, and the NDIT test dataset consisted of DDIs that two drugs were all in the drug test dataset. The model constructed on the training dataset was applied to two test datasets.

For convenience, the first cross-validation was called entire cross-validation, whereas the second one was termed composition cross-validation. The *K* was set to ten. The procedures of these two types of cross-validation are illustrated in Figure 1.

### 2.6. Performance Measurement

For a binary classification problem, the predicted results can be counted as four values, including true positive (TP), false positive (FP), true negative (TN), and false negative (FN). In detail, TP/TN represented the number of correctly predicted positive/negative samples, and FN/FP denoted the number of incorrectly predicted positive/negative samples. Based on these values, some measurements can be computed, such as precision, recall, accuracy, F1-measure, and the Mathews correlation coefficient (MCC) [36]. They can be computed by

(5) $$\begin{array}{c} \text{Precision}=\frac{\text{TP}}{\text{TP}+\text{FP}}, \end{array}$$

(6) $$\begin{array}{c} \text{Recall}=\frac{\text{TP}}{\text{TP}+\text{FN}}, \end{array}$$

(7) $$\begin{array}{c} \text{Accuracy}=\frac{\text{TP}+\text{TN}}{\text{TP}+\text{TN}+\text{FP}+\text{FN}}, \end{array}$$

(8) $$\begin{array}{c} \text{F}1‐\text{measure}=\frac{2\times \text{Precision}\times \text{Recall}}{\text{Precision}+\text{Recall}}=\frac{2\times \text{TP}}{2\times \text{TP}+\text{FN}+\text{FP}}, \end{array}$$

(9) $$\begin{array}{c} \text{MCC}=\frac{\text{TP}\times \text{TN}‐\text{FP}\times \text{FN}}{\sqrt{\left(\text{TN}+\text{FN}\right)\times \left(\text{TN}+\text{FP}\right)\times \left(\text{TP}+\text{FN}\right)\times \left(\text{TP}+\text{FP}\right)}}. \end{array}$$

The first four measurements were between 0 and 1, and high values meant high performance. The last measurement, MCC, ranged between -1 and 1, where 1 indicated perfect prediction and -1 suggested absolute wrong prediction.

In addition, to fully evaluate the performance of classifiers under different thresholds, the receiver operating characteristic (ROC) and precision-recall (PR) curve analyses were conducted. Given a threshold for predicting positive samples, the true positive rate (TPR) and false positive rate (FPR) can be computed, where TPR was the same as recall and FPR can be computed by

(10) $$\begin{array}{c} \text{FPR}=\frac{\text{FP}}{\text{TN}+\text{FP}}. \end{array}$$

After setting a series of thresholds, a group of TPR and FPR can be obtained. The ROC curve was plotted by setting TPR as the *y*-axis and FPR as the *x*-axis. The definition of the PR curve was similar to the ROC curve. It set precision as the *y*-axis and recall as the *x*-axis. The areas under these two curves were important measurements to assess the performance of classifiers. They were called AUROC and AUPR in this study.

## 3. Results and Discussion

In this study, a simple classifier using widely used fingerprints of drugs was proposed to predict DDIs. The whole procedure is illustrated in Figure 2. Here, detailed evaluation results were provided.

### 3.1. Performance of Classifiers under the Entire Tenfold Cross-Validation

Based on fingerprint features of drugs, three models were designed to generate three feature types of DDIs. By combining one or more feature types produced by different models, seven representations of DDIs were obtained, which were learnt by RF, respectively, to construct RF classifiers. Each classifier was evaluated by the entire tenfold cross-validation. Predicted results were counted as measurements calculated by Equations (5)–(9), which are listed in Table 1. It can be observed that classifiers using different combinations of feature types almost provided similar performance, except for the classifier using features produced by the Hadamard model. Relatively speaking, the classifier using features generated by addition and subtraction models and the classifiers using features produced by all three models were better than other classifiers. The classifier using features generated by addition and subtraction models provided the highest performance on precision, F1-measure, and MCC, whereas the classifiers using features produced by all three models yielded the best performance on accuracy and recall.

To further evaluate the performance of the above RF classifiers, the ROC and PR curves for each classifier were plotted, as shown in Figure 3. The key measurements AUROC and AUPR are also listed in this figure. Evidently, the classifier using features derived from the Hadamard model still provided the lowest AUROC and AUPR, whereas other classifiers yielded similar values on these two measurements. By careful comparisons, the classifier using features generated by addition and subtraction models provided the highest AUROC and AUPR, 0.9629 and 0.9601, respectively. Thus, it is believed that the classifier using features generated by addition and subtraction models was better than the classifier using features produced by all three models.

With the above arguments, we can construct the RF classifier using features generated by addition and subtraction models to predict DDIs. This classifier provided good performance under the entire tenfold cross-validation. It can be used to discover novel DDIs among known drugs.

### 3.2. Performance of Classifiers under Composition Tenfold Cross-Validation

In addition to the entire tenfold cross-validation, we also used composition tenfold cross-validation to assess RF classifiers using different combinations of feature types. As this cross-validation test involved two test datasets, including ODIT and NDIT test datasets, two groups of predicted results can be obtained, which are listed in Table 2. For the ODIT test dataset, the classifier using features produced by the Hadamard model was still evidently inferior to other classifiers. However, when adding the features yielded by the addition model, the classifier became much better, which provided the highest accuracy, precision, F1-measure, and MCC. The classifier using features generated by all models produced the highest recall. Accordingly, it can be concluded that the classifier using features obtained by the addition and Hadamard models gave the best performance on the ONIT test dataset. To further confirm this conclusion, the ROC and PR curves of seven classifiers were plotted, as shown in Figures 4(a) and 4(b). The classifier using features obtained by addition and Hadamard models yielded the highest AUROC (0.9026) and AUPR (0.8890). Thus, this classifier was better than other classifiers under such a test. Furthermore, it is easy to see that all measurements on the ODIT test dataset under the composition tenfold cross-validation were much lower than those under the entire tenfold cross-validation. For example, the MCC decreased by about 8%-20%. As one drug was not included in the training procedures, it was reasonable that the performance declined.

As for the NDIT test dataset, we also calculated five measurements described in Equations (5)–(9), which are also listed in Table 2. It can be observed that the highest value for each measurement was dispersive. The classifier using features obtained by addition and Hadamard models yielded the highest accuracy and MCC. Furthermore, from the ROC and PR curves on the NDIT test dataset, shown in Figures 4(c) and 4(d), such a classifier produced the highest AUROC and second-highest AUPR. Thus, we still concluded that such a classifier was best under such a test. Compared with the predicted results on the ODIT test dataset, those on NDIT were much lower. As two drugs were all not included in the training procedures, the performance was further declined.

In this section, we tested the classifiers under the composition tenfold cross-validation. Such a test was more rigid than the entire tenfold cross-validation because less information of the test sample was included in the training procedures. With the above arguments, the classifier using features obtained by the addition and Hadamard models was best, which can be a tool for predicting DDIs between known and unknown drugs or among unknown drugs.

### 3.3. Comparison of Classifiers Based on Support Vector Machine

We used RF to build the classifier for the prediction of DDIs. In fact, another classic classification algorithm, SVM [37], was also adopted to construct the classifier. The SVM program was also retrieved from scikit-learn. The kernel was a polynomial function, and the regularization parameter *C* was set to one. Here, we would elaborate that RF was more proper to build the efficient classifier.

For the best RF classifier under the entire tenfold cross-validation, it adopted the features generated by addition and subtraction models. The SVM classifier was also built by learning such representation of DDIs. The entire tenfold cross-validation was used to assess this SVM classifier. Obtained measurements, including accuracy, precision, recall, F1-measure, and MCC, are listed in Table 3. For easy comparison, the measurements yielded by the RF classifier are also provided in this table. It can be observed that the accuracy, precision, recall, and F1-measure were about 7% lower than those of the RF classifier, whereas the MCC was about 15% lower, indicating the superiority of the RF classifier. Furthermore, the ROC and PR curve analyses were also performed for this SVM classifier, as shown in Figures 5(a) and 5(b). Clearly, the SVM classifier provided lower AUROC and AUPR, further confirming the superiority of the RF classifier.

As for the best RF classifier under the composition tenfold cross-validation, the features generated by the addition and Hadamard models were used. The SVM classifier was also built on such representation of DDIs and evaluated by composition tenfold cross-validation. The predicted results on ODIT and NDIT test datasets are listed in Table 3. Likewise, the results of the RF classifier are also provided in this table for easy comparison. On the ODIT test dataset, the RF classifier was greatly superior to SVM classifier. All measurements were 10% higher, even 30% higher for MCC. Furthermore, as shown in Figures 5(c) and 5(d), the ROC and PR curves of the SVM classifier were always under those of the RF classifier, inducing lower AUROC and AUPR. This argument further confirmed the superiority of the RF classifier on the ODIT test dataset. On the NDIT test dataset, the performance of the SVM classifier was also lower than that of the RF classifier. For example, MCC was about 17% lower. However, the inferiority was smaller than that in the above tests. The SVM classifier even provided a higher performance on precision. The ROC and PR curves, shown in Figures 5(e) and 5(f), display a similar phenomenon, i.e., the SVM classifier yielded lower AUROC and AUPR. Thus, the RF classifier also provided a better performance on the NDIT test dataset than the SVM classifier.

Based on the above arguments, the RF classifier was always better than the SVM classifier no matter which cross-validation was adopted. It was reasonable to select RF for building the classifier.

### 3.4. Comparison of Classifiers Using Other Drug Features

Although the proposed RF classifier only adopted the drug fingerprint features, its performance was satisfied. To further elaborate on the utility of such a classifier, some classifiers using other drug features were constructed and compared with our classifier. To distinguish our classifier and other classifiers, we called our classifier a fingerprint-based classifier in this section.

The fingerprint-based classifier used the features derived from the binary fingerprint features of drugs. It was deemed to be a simple way. Some advanced schemes can be adopted to generate deep features of drugs. Here, we employed the natural language processing (NLP) method to produce drug features. First, 10763 drugs were retrieved from DrugBank, together with their SMILES. Second, the Morgan fingerprints [26] of these drugs were extracted by RDKit. 26932 substructures were obtained. Third, these substructures were termed words, and each drug was represented by these words. Such representation was fed into a NLP method, Word2vec [38], to generate the features of substructures. Finally, for a drug, the feature vectors of its substructures were collected, and their average vector was computed as the feature vector of the drug. Such obtained features were called text features. Based on these features, we generated two representations of DDIs. The first representation used the addition and subtraction models, and the second representation adopted the addition and Hadamard models, which were the best models of the fingerprint-based classifier under the entire and composition tenfold cross-validation, respectively. As the text features were not available for some drugs, we excluded these drugs and corresponding DDIs. Accordingly, the new dataset containing 26309 DDIs (positive samples) and the same number of drug pairs (negative samples) was constructed. Two RF classifiers with the above-mentioned two representations of DDIs were built on such dataset and evaluated by the corresponding tenfold cross-validation. These classifiers were called text-based classifiers. Also, fingerprint-based classifiers were also built and compared with text-based classifiers. The performance of fingerprint-based and text-based classifiers is listed in Table 4 and Figure 6. Under the entire tenfold cross-validation, the fingerprint-based classifier provided a much higher performance on all measurements. The same results occurred under the composition tenfold cross-validation on the ODIT test dataset. For the composition tenfold cross-validation on the NDIT test dataset, the fingerprint-based classifier provided higher values on recall, AUROC, and AUPR, but lower values on other measurements, suggesting the equal performance of these two classifiers. On the whole, the fingerprint-based classifier was superior to the text-based classifier. Although the fingerprint-based classifier used the drug features generated in a simple way, its performance was not low at all.

In recent years, a network is deemed to be a good form to organize research objects. To date, several studies adopted a network to investigate various drug-related problems [29, 39, 40]. The hidden information in one or more drug networks was quite different from that extracted from a single drug, giving a new view to investigate drugs. Here, we adopted the drug associations reported in STITCH [41] and KEGG [42] (SIMCOMP and SUBCOMP [43]) to construct three drug networks, where 772 drugs were defined as nodes and obtained associations were defined as edges. From these three networks, we adopted the scheme in a well-known network embedding method, Node2vec [44], to produce lots of paths. These paths were deemed as sentences, and nodes in paths were considered words, which were fed into Word2vec [38] to generate drug features. These features were called network features. Likewise, not all 772 drugs had network features as some drugs were isolated in all three networks. These drugs were excluded, and corresponding DDIs were also discarded. 3893 DDIs were accessed, which were put into a new dataset as positive samples. We also generated the same number of drug pairs, termed negative samples, and put them into such a new dataset. Then, two RF classifiers were built on such a dataset. One classifier adopted the features of DDIs derived from network features via addition and subtraction models, and the other classifier used the features of DDIs derived from network features using the addition and Hadamard models. The former classifier was evaluated by the entire tenfold cross-validation, and the late one was assessed by the composition tenfold cross-validation. For convenience, these classifiers were called a network-based classifier. For a fair comparison, two fingerprint-based classifiers were also built on the above-mentioned dataset. The performance of fingerprint-based and network-based classifiers is shown in Table 5 and Figure 7. Evidently, the fingerprint-based classifier was superior to the network-based classifier under the entire tenfold cross-validation. For the composition tenfold cross-validation on the ODIT test dataset, we can obtain the same result. As the results of the composition tenfold cross-validation on the NDIT test dataset, the superiority of the fingerprint-based classifier was not very obvious. On some measurements, the network-based classifier provided higher performance. However, this cannot prevent us from reaching the conclusion that the fingerprint-based classifier was superior to the network-based classifier.

With the above arguments, the fingerprint-based classifier was better than classifiers using features generated by some advanced computational methods. The simple representation scheme of the fingerprint-based classifier not only made the classifier easy to implement but also provided a satisfactory performance.

### 3.5. User Guide of the Web-Server

In this study, a RF classifier only using drug fingerprint features was proposed to predict DDIs. For wide applications of such a classifier, a web-server, named DDIPF, was set up. Users can access such web-server at http://106.14.164.77:5004/DDIPF/. The home page is illustrated in Figure 8.

Three tabs “Read Me,” “Supporting Information,” and “Citation” lie at the top of the home page. The basic information of this web-server can be found by clicking the “Read Me” button. Through the “Supporting Information” button, users can download the DDIs (positive samples) used in this study. The reference of this web-server is listed behind the “Citation” button.

Users can test the interaction probability of two drugs using the following steps:

Step1: input the SMILES formats of two drugs at the input boxes. Three examples can be found by clicking the “Example” button above the input boxes.

Step2: select one model or combination of two or more models at the drop-down box beside the “Feature model.” This can determine the representations of input drug pairs.

Step3: click the “Submit” button to upload the input drug pair.

Step4: after a few seconds, the probability is displayed in the box beside the “The probability is.” A high probability indicates two input drugs can interact with high likelihood. Users can click the “Clear” button for another input.

## 4. Conclusions

This study proposed a simple classifier to predict drug-drug interactions. The classifier only adopted the widely used fingerprint features of drugs, which induced it to have wider applications than most previous methods. On the other hand, the classifier provided good performance when one or two drugs in the DDI were used in the training procedure, indicating that it can be a latent tool to predict possible drug-drug interactions. However, if two drugs in the DDI were not included in the training procedure, the classifier was not good enough. In the future, we will improve the classifier in this regard. Furthermore, we set up a web-server (http://106.14.164.77:5004/DDIPF/). Users can easily test drug pairs through such web-server. We hope this contribution can improve the research on drug-drug interactions.

## Figures and Tables

**Figure 1:** Procedures of two types of cross-validation. (a) Entire cross-validation; (b) Composition cross-validation.

**Figure 2:** Whole construction procedures of the classifier for predicting drug-drug interactions (DDIs). Validated DDIs are retrieved from DrugBank, which are termed positive samples. Drugs involved in positive samples are used to randomly generate negative samples. Drugs are represented by fingerprint features, which are further refined as DDI features using three models. Random forest is adopted to build the classifier, which is evaluated by two types of tenfold cross-validation.

**Figure 3:** Performance of the classifiers using different combinations of feature types under the entire tenfold cross-validation evaluated by ROC and PR curves. (a) ROC curves. (b) PR curves.

**Figure 4:** Performance of the classifiers using different combinations of feature types under the composition tenfold cross-validation evaluated by ROC and PR curves. (a) The ROC curves on the ODIT test dataset. (b) The PR curves on the ODIT test dataset. (c) ROC curves on the NDIT test dataset. (d) The PR curves on the NDIT test dataset.

**Figure 5:** Performance of the RF and SVM classifiers under two types of tenfold cross-validation evaluated by ROC and PR curves. (a) The ROC curve under the entire tenfold cross-validation. (b) The PR curve under the entire tenfold cross-validation. (c) The ROC curve on the ODIT test dataset under the composition tenfold cross-validation. (d) The PR curve on the ODIT test dataset under the composition tenfold cross-validation. (e) The ROC curve on the NDIT test dataset under the composition tenfold cross-validation. (f) The PR curve on the NDIT test dataset under the composition tenfold cross-validation.

**Figure 6:** Performance of the fingerprint- and text-based classifiers (random forest) under two types of tenfold cross-validation evaluated by the ROC and PR curves. (a) The ROC curve under the entire tenfold cross-validation; (b) the PR curve under the entire tenfold cross-validation; (c) the ROC curve on the ODIT test dataset under the composition tenfold cross-validation; (d) the PR curve on the ODIT test dataset under the composition tenfold cross-validation; (e) the ROC curve on the NDIT test dataset under the composition tenfold cross-validation; (f) the PR curve on the NDIT test dataset under the composition tenfold cross-validation.

**Figure 7:** Performance of the fingerprint- and network-based classifiers (random forest) under two types of tenfold cross-validation evaluated by the ROC and PR curves. (a) The ROC curve under the entire tenfold cross-validation; (b) the PR curve under the entire tenfold cross-validation; (c) the ROC curve on the ODIT test dataset under the composition tenfold cross-validation; (d) the PR curve on the ODIT test dataset under composition tenfold cross-validation; (e) the ROC curve on the NDIT test dataset under the composition tenfold cross-validation; (f) the PR curve on the NDIT test dataset under the composition tenfold cross-validation.

**Figure 8:** Homepage of the web-server DDIPF.

**Table 1:** Performance of RF classifiers with different combinations of feature types under the entire tenfold cross-validation^#^.

Model	Accuracy	Precision	Recall	F1-measure	MCC^a^
Addition	89.26%	92.53%	86.85%	89.60%	78.69%
Subtraction	88.84%	*92.31%*	86.32%	*89.22%*	77.88%
Hadamard	73.63%	74.71%	73.13%	73.91%	47.27%
Addition + subtraction	89.33%	92.70%	87.20%	89.86%	*79.25%*
Addition + Hadamard	88.51%	92.14%	86.64%	89.30%	78.09%
Subtraction + Hadamard	88.81%	92.01%	86.48%	89.16%	77.78%
Addition + subtraction + Hadamard	*89.47%*	92.34%	*87.33%*	89.76%	79.08%

^#^Numbers in italics indicate the highest values in the corresponding column. ^a^The Mathews correlation coefficient.

**Table 2:** Performance of RF classifiers with different combinations of feature types under the composition tenfold cross-validation^#^.

Test set	Model	Accuracy	Precision	Recall	F1-measure	MCC^a^
ODIT^b^ test dataset	Addition	79.62%	74.27%	83.18%	78.46%	59.61%
	Subtraction	78.60%	72.65%	82.46%	77.23%	57.63%
	Hadamard	69.19%	65.84%	70.56%	68.10%	38.49%
	Addition + subtraction	79.07%	72.71%	83.32%	77.63%	58.65%
	Addition + Hadamard	*79.86%*	*75.20%*	82.99%	*78.89%*	*60.06%*
	Subtraction + Hadamard	79.63%	74.74%	82.84%	78.57%	59.56%
	Addition + subtraction + Hadamard	79.39%	73.49%	*83.33%*	78.08%	59.21%
NDIT^c^ test dataset	Addition	63.58%	37.60%	*78.53%*	50.56%	31.88%
	Subtraction	63.56%	39.66%	76.27%	52.01%	30.99%
	Hadamard	62.40%	*54.91%*	64.56%	*59.21%*	25.15%
	Addition + subtraction	63.41%	37.72%	77.78%	50.50%	31.34%
	Addition + Hadamard	*64.49%*	41.56%	76.82%	53.73%	32.64%
	Subtraction + Hadamard	64.39%	42.04%	76.18%	53.99%	32.26%
	Addition + subtraction + Hadamard	63.92%	39.72%	77.16%	52.21%	31.88%

^#^Numbers in italics indicate the highest values in the corresponding column. ^a^MCC: Mathews correlation coefficient. ^b^ODIT: One Drug In Train set. ^c^NDIT: No Drug In Train set.

**Table 3:** Comparison of RF and SVM classifiers under the two types of tenfold cross-validation.

Cross-validation		Classification algorithm	Model	Accuracy	Precision	Recall	F1-measure	MCC^a^
Entire tenfold cross-validation		Random forest	Addition + subtraction	89.54%	92.70%	87.20%	89.86%	79.25%
		Support vector machine		81.92%	85.92%	79.57%	82.62%	64.06%
Composition tenfold cross-validation	ODIT^b^ test dataset	Random forest	Addition + Hadamard	79.86%	75.20%	82.99%	78.89%	60.06%
		Support vector machine		64.65%	61.20%	65.53%	63.06%	29.51%
	NDIT^c^ test dataset	Random forest	Addition + Hadamard	64.49%	41.56%	76.82%	53.73%	32.64%
		Support vector machine		57.45%	48.26%	58.41%	52.46%	15.07%

^a^MCC: Mathews correlation coefficient. ^b^ODIT: One Drug In Train set. ^c^NDIT: No Drug In Train set.

**Table 4:** Comparison of fingerprint- and text-based classifiers under two types of tenfold cross-validation.

Cross-validation		Classifier	Model	Accuracy	Precision	Recall	F1-measure	MCC^a^
Entire tenfold cross-validation		Fingerprint-based classifier (random forest)	Addition + subtraction	89.55%	92.25%	87.53%	89.83%	79.23%
		Text-based classifier (random forest)		84.16%	87.52%	82.01%	84.67%	68.48%
Composition tenfold cross-validation	ODIT^b^ test dataset	Fingerprint-based classifier (random forest)	Addition + Hadamard	80.01%	75.80%	82.81%	79.07%	60.33%
		Text-based classifier (random forest)		77.55%	72.92%	80.37%	76.42%	55.39%
	NDIT^c^ test dataset	Fingerprint-based classifier (random forest)	Addition + Hadamard	65.06%	42.58%	77.55%	54.49%	33.81%
		Text-based classifier (random forest)		66.97%	54.38%	72.80%	61.73%	35.26%

^a^Mathews correlation coefficient. ^b^ODIT: One Drug In Train set. ^c^NDIT: No Drug In Train set.

**Table 5:** Comparison of fingerprint- and network-based classifiers under two types of tenfold cross-validation.

Cross-validation		Classifier	Model	Accuracy	Precision	Recall	F1-measure	MCC^a^
Entire tenfold cross-validation		Fingerprint-based classifier (random forest)	Addition + subtraction	86.86%	89.21%	85.23%	87.16%	73.82%
		Network-based classifier (random forest)		77.88%	77.60%	78.06%	77.81%	55.79%
Composition tenfold cross-validation	ODIT^b^ test dataset	Fingerprint-based classifier (random forest)	Addition + Hadamard	74.31%	72.43%	75.46%	73.77%	48.83%
		Network-based classifier (random forest)		70.79%	66.72%	72.65%	69.31%	41.94%
	NDIT^c^ test dataset	Fingerprint-based classifier (random forest)	Addition + Hadamard	59.99%	33.23%	70.80%	43.48%	23.34%
		Network-based classifier (random forest)		57.53%	41.20%	62.17%	48.49%	16.42%

^a^Mathews Correlation Coefficient. ^b^ODIT: One Drug In Train set. ^c^NDIT: No Drug In Train set.

## Data Availability

The original data used to support the findings of this study are available in the DrugBank database.

## References

[1] Lee G., Park C., Ahn J. (2019). Novel deep learning model for more accurate prediction of drug-drug interaction effects. *BMC Bioinformatics*.

[2] Percha B., Altman R. B. (2013). Informatics confronts drug-drug interactions. *Trends in Pharmacological Sciences*.

[3] Becker M. L., Kallewaard M., Caspers P. W. J., Visser L. E., Leufkens H. G. M., Stricker B. H. C. (2007). Hospitalisations and emergency department visits due to drug–drug interactions: a literature review. *Pharmacoepidemiology and Drug Safety*.

[4] Wishart D. S., Knox C., Guo A. C. (2006). DrugBank: a comprehensive resource for in silico drug discovery and exploration. *Nucleic Acids Research*.

[5] Wishart D. S., Knox C., Guo A. C. (2008). DrugBank: a knowledgebase for drugs, drug actions and drug targets. *Nucleic Acids Research*.

[6] Kanehisa M., Furumichi M., Tanabe M., Sato Y., Morishima K. (2017). KEGG: new perspectives on genomes, pathways, diseases and drugs. *Nucleic Acids Research*.

[7] Kuhn M., Szklarczyk D., Pletscher-Frankild S. (2014). STITCH 4: integration of protein–chemical interactions with user data. *Nucleic Acids Research*.

[8] Yan C., Duan G., Pan Y., Wu F. X., Wang J. (2019). DDIGIP: predicting drug-drug interactions based on Gaussian interaction profile kernels. *BMC Bioinformatics*.

[9] Kastrin A., Ferk P., Leskosek B. (2018). Predicting potential drug-drug interactions on topological and semantic similarity features using statistical learning. *PLoS One*.

[10] Cheng F. X., Zhao Z. M. (2014). Machine learning-based prediction of drug-drug interactions by integrating drug phenotypic, therapeutic, chemical, and genomic properties. *Journal of the American Medical Informatics Association*.

[11] Chen L., Chu C., Zhang Y. H. (2017). Identification of drug-drug interactions using chemical interactions. *Current Bioinformatics*.

[12] Gottlieb A., Stein G. Y., Oron Y., Ruppin E., Sharan R. (2012). INDI: a computational framework for inferring drug interactions and their associated recommendations. *Molecular Systems Biology*.

[13] Cami A., Manzi S., Arnold A., Reis B. Y. (2013). Pharmacointeraction network models predict unknown drug-drug interactions. *PLoS One*.

[14] Liu S. Y., Tang B., Chen Q., Wang X. (2016). Drug-drug interaction extraction via convolutional neural networks. *Computational and Mathematical Methods in Medicine*.

[15] Sun X., Dong K., Ma L. (2019). Drug-drug interaction extraction via recurrent hybrid convolutional neural networks with an improved focal loss. *Entropy*.

[16] Zhang Y., Qiu Y., Cui Y., Liu S., Zhang W. (2020). Predicting drug-drug interactions using multi-modal deep auto-encoders based network embedding and positive-unlabeled learning. *Methods*.

[17] Fatehifar M., Karshenas H. (2021). Drug-drug interaction extraction using a position and similarity fusion-based attention mechanism. *Journal of Biomedical Informatics*.

[18] Huang J., Niu C., Green C. D., Yang L., Mei H., Han J. D. J. (2013). Systematic prediction of pharmacodynamic drug-drug interactions through protein-protein-interaction network. *PLoS Computational Biology*.

[19] Guimera R., Sales-Pardo M. (2013). A network inference method for large-scale unsupervised identification of novel drug-drug interactions. *PLoS Computational Biology*.

[20] Takarabe M., Shigemizu D., Kotera M., Goto S., Kanehisa M. (2011). Network-based analysis and characterization of adverse drug–drug interactions. *Journal of Chemical Information and Modeling*.

[21] Liu N., Chen C. B., Kumara S. (2020). Semi-supervised learning algorithm for identifying high-priority drug–drug interactions through adverse event reports. *IEEE Journal of Biomedical and Health Informatics*.

[22] Asada M., Miwa M., Sasaki Y. (2020). Using drug descriptions and molecular structures for drug–drug interaction extraction from literature. *Bioinformatics*.

[23] Shen Y., Yuan K., Yang M. (2019). KMR: knowledge-oriented medicine representation learning for drug–drug interaction and similarity computation. *Journal of Cheminformatics*.

[24] Breiman L. (2001). Random forests. *Machine Learning*.

[25] Weininger D. (1988). SMILES, A chemical language and information system. 1. Introduction to methodology and encoding rules. *Journal of Chemical Information and Computer Sciences*.

[26] Rogers D., Hahn M. (2010). Extended-connectivity fingerprints. *Journal of Chemical Information and Modeling*.

[27] Wang Y., Xu Y., Yang Z., Liu X., Dai Q. (2021). Using recursive feature selection with random forest to improve protein structural class prediction for low-similarity sequences. *Computational and Mathematical Methods in Medicine*.

[28] Chen W., Chen L., Dai Q. (2021). iMPT-FDNPL: identification of membrane protein types with functional domains and a natural language processing approach. *Computational and Mathematical Methods in Medicine*.

[29] Yang Y., Chen L. (2022). Identification of drug–disease associations by using multiple drug and disease networks. *Current Bioinformatics*.

[30] Baranwal M., Magner A., Elvati P., Saldinger J., Violi A., Hero A. O. (2020). A deep learning architecture for metabolic pathway prediction. *Bioinformatics*.

[31] Carlos M., Zoran K., Juan S. (2021). Predicting non-deposition sediment transport in sewer pipes using random forest. *Water Research*.

[32] Casanova R., Saldana S., Chew E. Y., Danis R. P., Greven C. M., Ambrosius W. T. (2014). Application of random forests methods to diabetic retinopathy classification analyses. *PLoS One*.

[33] Fernandez-Delgado M., Cernadas E., Barro S., Amorim D. (2014). Do we need hundreds of classifiers to solve real world classification problems?. *Journal of Machine Learning Research*.

[34] Pedregosa F., Varoquaux G., Gramfort A. (2011). Scikit-learn: machine learning in python. *Journal of Machine Learning Research*.

[35] Kohavi R. (1995). A Study of Cross-Validation and Bootstrap for Accuracy Estimation and Model Selection.

[36] Matthews B. (1975). Comparison of the predicted and observed secondary structure of T4 phage lysozyme. *Structure*.

[37] Cortes C., Vapnik V. (1995). Support-vector networks. *Machine Learning*.

[38] Church K. W. (2017). Word2Vec. *Natural Language Engineering*.

[39] Luo Y., Zhao X., Zhou J. (2017). A network integration approach for drug-target interaction prediction and computational drug repositioning from heterogeneous information. *Nature Communications*.

[40] Zhou J.-P., Chen L., Guo Z.-H. (2020). iATC-NRAKEL: an efficient multi-label classifier for recognizing anatomical therapeutic chemical classes of drugs. *Bioinformatics*.

[41] Kuhn M., von Mering C., Campillos M., Jensen L. J., Bork P. (2007). STITCH: interaction networks of chemicals and proteins. *Nucleic Acids Research*.

[42] Kanehisa M., Goto S. (2000). KEGG: Kyoto Encyclopedia of Genes and Genomes. *Nucleic Acids Research*.

[43] Hattori M., Tanaka N., Kanehisa M., Goto S. (2010). SIMCOMP/SUBCOMP: chemical structure search servers for network analyses. *Nucleic Acids Research*.

[44] Grover A., Leskovec J. node2vec: scalable feature learning for networks.

